# Bidirectional Effect of Repeated Exposure to Extremely Low-Frequency Electromagnetic Field (50 Hz) of 1 and 7 mT on Oxidative/Antioxidative Status in Rat's Brain: The Prediction for the Vulnerability to Diseases

**DOI:** 10.1155/2022/1031211

**Published:** 2022-06-14

**Authors:** Angelika Klimek, Anna Nowakowska, Hanna Kletkiewicz, Joanna Wyszkowska, Justyna Maliszewska, Milena Jankowska, Lukasz Peplowski, Justyna Rogalska

**Affiliations:** ^1^Department of Animal Physiology and Neurobiology, Faculty of Biological and Veterinary Sciences, Nicolaus Copernicus University in Torun, 87-100, Poland; ^2^Department of Biophysics, Institute of Physics, Faculty of Physics, Astronomy and Informatics Nicolaus Copernicus University in Torun, 87-100, Poland

## Abstract

Studies reported evidence for opposite effects of extremely low-frequency electromagnetic field (EMF): harmful, including the oxidative stress induction, and beneficial, such as the activation of antioxidant defense. People's exposure to EMF is often repeated or prolonged, and it is important to consider the cumulative effect of such kind of exposure on the organism. If changes evoked by repeated exposure to EMF are permanent, responsiveness to other stress factors can be modified. The aims of our study were (1) to evaluate changes in the levels of oxidative stress and antioxidant defense markers in the prefrontal cortex of adult rats after repeated exposure to 1 and 7 mT EMF and (2) to assess whether repeated EMF exposure can modify oxidative/antioxidative status in response to other stress factors. Rats were exposed to EMF 1 h/day for 7 days, one, twice, or three times. After each exposure, 8-isoprostanes, protein carbonyl groups, and the total antioxidant capacity were assessed. Part of the animals, after EMF treatment, was exposed to another stress factor—open field. Results showed that repeated exposure changed the oxidative/antioxidative status depending on the intensity of the EMF and the number of exposures. 1 mT EMF created weak changes in the oxidative status in the brain; however, 7 mT EMF moved the balance to a clearly higher level. The changes in the oxidative status after 1 mT EMF were enough to reduce, and after 7 mT EMF to intensify oxidative processes in response to the next stress. We concluded that the organism might adapt to “weak” EMF, while “strong” EMF exceeds the adaptive capacity of the organism and sensitizes it to subsequent stress, and thus may modulate vulnerability to diseases. Our results also provide new insights into the possible therapeutic properties of the magnetic field, as 1 mT EMF appears to have a potentially protective impact on the brain.

## 1. Introduction

The influence of the extremely low-frequency electromagnetic field (EMF) on living organisms is still being widely investigated. EMF includes frequencies in the range of 3-300 Hz, which also correspond to physiological brain oscillations [1]. The most common frequencies values in our environment are 50 Hz and 60 Hz [2, 3]. Nowadays, people are increasingly exposed to this type of electromagnetic field due to the increasing number of electrical devices in our urbanized environment. EMF exposure has been proved to be an important risk factor in the development of diseases affecting the nervous system, such as anxiety or depression [4]. The brain is an organ extremely sensitive to oxidative stress because of the high amount of unsaturated lipids, energetics dependent on mitochondria, neurotransmitters' metabolism generating hydrogen peroxide (H_2_O_2_), the ability of neurotransmitters to autooxidation, and engagement of reactive oxygen species in Ca^2+^ signaling [5]. Oxidative stress underlies many neurodegenerative and neuropsychiatric disorders [6].

The results of studies concerning the effect of EMF (50/60 Hz) on oxidative stress and antioxidant defense are often contradictory or insufficient. It means that the answer to the question whether EMF has a beneficial or detrimental impact on the organism is not obvious. Some authors reported evidence for the harmful effects of EMF, including oxidative stress induction [7–9]. The increased level of one of the most common markers of lipid peroxidation, malondialdehyde (MDA), was noticed in a several studies on humans and animal models exposed to EMF [7, 8]. In addition, oxidative damages are often accompanied by a decrease in antioxidant defense [8–10]. On the other hand, the increase of reports on the benefits associated with exposure to EMF such as activation of antioxidant systems is observed [11–13]. These protective effects of EMF are also used in medicine, e.g., for the treatment of brain damages [13]. It is also important that EMF exposure experienced by people is often repeated or prolonged, but most research evaluates the effect of the single period of EMF exposure.

EMF is recognized as a mild stress factor [2, 14], which as other stress factors can result in different activations of stress response systems; it means that exposure to EMF can establish a new “set-point” for stress systems activity. However, the course of this phenomenon (the direction and dynamics) depends on the intensity of the electromagnetic field. As a consequence, the EMF-induced changes in stress hormones can boost “cellular hormesis” by activation of signaling pathways including oxidative/antioxidative processes in different ways [15].

Here, we propose the hypothesis that the impact of an extremely low-frequency electromagnetic field on oxidant/antioxidant balance is not definitely negative, and the direction and dynamics of EMF-induced changes depend on the value of magnetic flux density as well as on the number of exposures. During repeated exposure to some stress factor, the organism responds to each individual stressor; however, consequently, the cumulative effect of all exposures is observed. As a result, temporary or permanent regulatory changes can be evoked [16]. The first exposure to stress generates the stress-induced initial disruption in homeostasis. As the response, the processes to reestablish the balance are triggered and they require gene expression and protein synthesis that progresses over time; thus, the temporal feature of the response to repetitive stress is essential [17]. We assumed that the first exposure to EMF changes the oxidative/antioxidative status; thus, each next EMF exposure would overlap its level established under the previous EMF exposure.

Therefore, the first aim of the study was to evaluate the changes in the levels of oxidative stress as well as the antioxidant defense markers in the prefrontal cortex of adult rats after repeated exposure to EMF of two different values of magnetic flux density (1 and 7 mT). The prefrontal cortex seems to be more sensitive to oxidative stress than other brain structures and concerning its role in the development of nervous system-related diseases; it appears to be relevant for research of the impact of EMF on oxidative/antioxidative status [18]. We have chosen to evaluate the effects of EMF of 1 and 7 mT. According to European Union Directive 2013/35/EU, the threshold value for magnetic flux density of the minor transient changes in the brain is set to a value of 1 mT EMF for 50 Hz. On the other hand, the exposure of workers to 50 Hz magnetic fields must be limited to the value 6 mT [19]. It has been shown that exposure to EMF of intensity higher than 6 mT causes measurable biological effects, e.g., increased lipid peroxidation [20, 21], DNA damage [22], and neuronal networks synchrony firing generation [23].

Then, we assumed that if the changes evoked by repeated exposure to EMF are permanent, the responsiveness to the other kinds of stress can be modified. It means that EMF can change the vulnerability of the organism to subsequent stress factors and thus to diseases, mainly related to the nervous system, in a two-way manner: compensatory or detrimental ones. Intriguingly, many nervous system-related disorders may be accounted for by a ‘two-hit model' in which environmental stressors change the central nervous system function in the permanent way leading to changes in vulnerability to a “second hit,” in turn leading to the onset of disease [24]. Thus, the second aim of the research was to assess whether the consequence of repeated EMF exposure can be the modification of the oxidative/antioxidative status in response to subsequent, other stress factors.

## 2. Materials and Methods

### 2.1. Animals

A total of 175 male adults (3-month-old) Wistar rats weighing 300-350 g were used throughout the experimentation. The number of animals in the research was planned in accordance with 3R principles (replacement, reduction, and refinement; EU Directive 2010/63/EU) [25]. Rats were housed in plastic cages in a temperature/humidity/light-controlled laboratory conditions (22 ± 2°C, humidity 55 ± 10%, 12 : 12 h light : dark cycle with lights on at 7:00 a.m.). Rodent laboratory feed and drinking water were provided ad libitum. All experimental procedures were approved by the Local Committee for Ethics in Animal Research in Bydgoszcz, Poland (decision number: 3/2018).

### 2.2. In Vivo Electromagnetic Field Exposure System

Animals were exposed to 50 Hz sinusoidal electromagnetic field of 1 mT and 7 mT (root mean square (RMS)) flux density, generated in a coil of 0.1 m in radius, designed by EiE (Elektronika i Elektromedycyna Sp. J., Otwock, Poland). This exposure system has been described in detail previously [3, 26]. The EMF was regulated during exposure by input current to the coil, and the magnetic flux density was measured before each experiment with a Gauss meter (Model GM2, AlphaLab, Inc., USA). The nonhomogeneity of the EMF within the area containing the animal's cage was < 15% (Figure 1). The temperature during all experiments was monitored using thermocouples mounted in the animal cages, and it was set to 26 ± 1°C.

### 2.3. Experimental Design

One week after habituation to the laboratory environment, the rats in individual plastic cages (12 cm × 20 cm × 14 cm, with a perforated plexiglass cover and wood shavings bedding) were put into the centre of the EMF coil. Exposure to “low” (1 mT) and “high” (7 mT) EMF was performed for three periods described as *E*1, *E*2, and *E*3. Each period included 7-day exposure, 1 h/1day. Rats subjected to the same experimental procedure except electromagnetic field exposure were used as the control.

The experimental design included two sets of experiments (Figure 2). During the first set of experiments, a part of rats (*n* = 88) after each period of EMF or control exposure (*E*1, *E*2, and *E*3) was decapitated to estimate the effect of EMF on oxidant/antioxidant status (8-isoprostanes (8-epi PGF2*α*), protein carbonyl (CP) groups, and level of total antioxidant capacity (TAC)—described in this research as “basal” (B) level) (Figure 2(a)). The remaining rats from each group (*n* = 87) were used during the second set of experiments (Figure 2(b)). The experiments as previously included one to three periods of EMF or control exposure (*E*1, *E*2, or *E*3), and after each of them the part of animals was exposed to another kind of stress factor—open field (OF) (size of the box: 100 cm × 100 cm, duration of the test: 5 min). It is a stress-induced procedure (exposure to a novel, open, light environment), which was proved to evoke the activation of brain stress systems. Then, the animals were decapitated for assessment of stress-induced changes in oxidant/antioxidant parameters as a consequence of previous exposure to EMF. To avoid the influence of the circadian rhythm on the results, decapitation was performed between 10:00 and 12:00 am.

The rats were divided into six groups: (1) EMF/B/1mT: animals exposed to EMF (50 Hz, 1 mT), in which the basal (B) level of markers was assessed; (2) EMF/OF/1mT: animals exposed to EMF (50 Hz, 1 mT) and exposed to open field test (OF); (3) EMF/B/7mT: animals exposed to EMF (50 Hz, 7 mT) in which the basal (B) level of markers was assessed; (4) EMF/OF/7mT: animals exposed to EMF (50 Hz, 7 mT) and exposed to open field test (OF); (5) C/B: control animals subjected to the same experimental procedure as the experimental groups 1 and 3, except EMF exposure; (6) C/OF: control animals subjected to the same experimental procedure as the experimental groups 2 and 4, except EMF exposure.

### 2.4. Sample Collection

After decapitation, the part of the brain (prefrontal cortex) was quickly dissected. Each fragment of tissue was weighed and immediately frozen in liquid nitrogen and stored at −80°C until further biochemical analysis. For determination of oxidant/antioxidant status, brain samples were homogenized on ice in phosphate buffer pH 7.4. After centrifugation for 10 minutes at 12000 x g, the supernatants were collected in Eppendorf tubes and stored until they were used for the assessment of the level of protein carbonyl (CP) groups and 8-isoprostanes (8-epi PGF2*α*) as a result of proteins and phospholipid peroxidation, respectively, as well as the total nonenzymatic antioxidant capacity (TAC).

### 2.5. Determination of the Markers of Oxidant/Antioxidant Status Level

Protein carbonyl (CP) groups and 8-isoprostanes (8-epi PGF2*α*) as well as total nonenzymatic antioxidant capacity (TAC) concentrations were determined with commercial kits according to the manufacturers' instructions. Each sample was assayed in triplicate. Colorimetric changes in the assay were detected using a multimode microplate reader Epoch 2 (BioTek Instruments, Inc., Winooski, UT, USA).

#### 2.5.1. Determination of Protein Peroxidation

The level of end product of protein peroxidation-protein carbonyl (CP) groups was assayed using a Protein Carbonyl Content Assay Kit (Sigma-Aldrich, No MAK094, USA) based on their reaction with 2,4-dinitrophenylohydrazine (DNPH). Finally, dinitrophenyl (DNP) hydrazone adducts were formed and then were detected spectrophotometrically at 375 nm. The level of DNP was proportional to the concentrations of CP. The amount of carbonyl in the sample well was calculated per 1 mg of protein. Results were expressed as nanomoles per mg of protein.

#### 2.5.2. Determination of Phospholipid Peroxidation

The level of end product of phospholipid peroxidation–8-isoprostanes (8-epi PGF2*α*) was assayed using 8-isoprostane ELISA Kit (Cayman Chemical, No 516351, USA). 8-Isoprostane has been proposed as a marker of oxidative stress and antioxidant deficiency. Isoprostanes are prostaglandin (PG) isomers that are generated from polyunsaturated fatty acids, mainly from arachidonic acid by a nonenzymatic process that involves peroxidation of membrane phospholipids by free radicals and reactive oxygen species. The absorbance of samples was measured at 406 nm. The concentration of 8-epi PGF2*α* was expressed as picograms per milliliter of sample.

#### 2.5.3. Determination of Total Antioxidant Capacity

TAC was determined using a Total Antioxidant Capacity Assay Kit (Sigma-Aldrich, No MAK187, USA) in which concentrations of both small molecules and protein antioxidants were determined. Determination of TAC is based on reduction Cu^2+^ to Cu^+^ by both small molecules and proteins but using the Protein Mask prevents Cu^2+^ reduction by proteins. Finally, the amount of reduced Cu^+^ ion enabling the analysis of small molecule antioxidants. The reduced Cu^+^ ions chelate with a colorimetric probe. The absorbance (peak at 570 nm) is proportional to the TAC level in Trolox equivalents (a water-soluble vitamin E analogue used as an antioxidant standard). Results were calculated as nanomoles per milliliter of sample.

### 2.6. Data Analysis

To analyze the effect of repeated exposure to EMF on the markers of oxidative stress and total antioxidant capacity, we applied a general linear model (GLM) allowing to determine the effect of a combination of two fixed categorical factors: EMF intensity and number of exposures (1 mT, 7 mT vs. *E*1, *E*2, and *E*3). The levels of the open field-induced oxidative stress and antioxidant markers were compared to their basal levels for each group, respectively: C/B vs. C/OF, EMF/B/1mT vs. EMF/OF/1mT, and EMF/B/7mT vs. EMF/OF/7mT using GLM with open field/basal level and number of exposures as fixed categorical factors. If necessary the data were log-transformed after checking for normality (Shapiro-Wilk test) and homoscedasticity (Levene test). Differences between compared data were considered significant when *P* < 0.05. The analyses were carried out using SPSS 25.0 package (IBM Inc.).

## 3. Results

### 3.1. The Basal Level of Oxidative Stress Markers

#### 3.1.1. Protein Carbonyl (CP) Groups

The intensity of EMF, as well as the number of exposures, had an influence on the basal level of CP groups in the prefrontal cortex. The CP groups' level increased with increasing EMF intensity, and the subsequent exposures enhanced the effect. There was also a significant interaction between these two factors (Table 1(a), Figure 3(a)). After first (*E*1) and second exposures (*E*2) to EMF of 1 mT the level of CP groups in the rat's brain did not differ from the control level; however, CP level after *E*2 was significantly higher than that after *E*1 (*P* < 0.01). After the third exposure (*E*3), CP level increased significantly compared to the control group (*P* < 0.001) and was also significantly higher than that noticed after *E*1 (*P* < 0.001) and *E*2 (*P* < 0.01). In animals exposed to EMF of 7 mT after *E*1, we observed a slight elevation in the level of the CP groups in comparison to control values, after *E*2 as well as after *E*3; however, the increase in CP level was significant (*P* < 0.001). Moreover, the statistically significant increase in the CP level after *E*2 was observed in comparison to that observed after *E*1 (*P* < 0.01), whereas after *E*3, the CP level was not significantly different from the value determined after *E*2. In animals exposed to EMF of 7 mT, the level of CP was enhanced in comparison to the value in the EMF/B/1mT group after *E*1 and *E*2 (*P* < 0.001) and the difference disappeared after *E*3.

#### 3.1.2. 8-Isoprostanes (8-epi PGF2*α*)

The level of 8-epi PGF2*α* after exposure to EMF was dependent only on the strength of the electromagnetic field (Table 1(b), Figure 3(b)). The exposure to EMF of 1 mT did not significantly affect the level of 8-epi PGF2*α* regardless of the number of exposures. Also, the analysis showed no clear differences between values of this parameter observed after *E*1 to *E*3. However, the tendency to decrease in the level of 8-epi PGF2*α* with each subsequent exposure was observed (Figure 3(b)). Otherwise, in the EMF/B/7mT group, the tendency to increase in the level of 8-epi PGF2*α* with each next exposure was noticed (Figure 3(b)). After *E*3, the level of 8-epi PGF2*α* was clearly higher in the group exposed to EMF of 7 mT compared to the control group as well as to that in the EMF/B/1mT group (*P* < 0.001).

### 3.2. The Open Field-Induced Level of Oxidative Stress Markers

#### 3.2.1. Protein Carbonyl (CP) Groups

The direction of changes in CP level in animals exposed to EMF of 1 mT and 7 mT after exposure to subsequent stress factor—open field test (EMF/OF/1mT and EMF/OF/7mT groups) coincided with their basal level observed only after exposure to electromagnetic field (EMF/B/1mT and EMF/B/7mT groups). Both intensity of the EMF and the number of exposures had an effect on the open field-induced level of CP groups. The interaction of both factors was also significant (Table 1(c), Figure 4(a)). There were no significant differences between the EMF/OF/1mT and C/OF groups after *E*1 and *E*2, but after *E*3 the level of CP in the group exposed to EMF of 1 mT was even lower in comparison to the value in the respective control group (C/OF) (*P* < 0.001). After a single exposure to EMF of 1 mT, the CP level was higher than that noticed after *E*2 and *E*3 (*P* < 0.001), while no significant difference was noticed between values after *E*2 and *E*3. The lowest value of CP groups in the EMF/OF/1mT group was observed after *E*3. The level of CP in the EMF/OF/7mT group was significantly increased compared to control animals after each exposure (*P* < 0.001) and was the highest after *E*3. The value observed after *E*2 was lower compared to both *E*1 and *E*3 (*P* < 0.001). Regardless of the number of exposures, the level of CP was always higher in the EMF/OF/7mT group in comparison to the values observed in the EMF/OF/1mT group (*P* < 0.001).

#### 3.2.2. 8-Isoprostanes (8-epi PGF2*α*)

The direction of OF-induced changes in the 8-epi PGF2*α* level was similar to that in the basal level of this marker. A significant impact of EMF intensity and the combination of two factors (EMF intensity x number of exposures) was noticed (Table 1(d); Figure 4(b)). There was no significant difference in 8-epi PGF2*α* level between the control group (C/OF) and animals exposed to EMF of 1 mT after *E*1; however, the level of this parameter after *E*2 was decreased compared to the control value (*P* < 0.05), and after *E*3, it returned to the control value. The decrease in 8-epi PGF2*α* level was also observed after *E*2 relative to *E*1 (*P* < 0.05). In the EMF/OF/7mT group, the clear increase of 8-epi PGF2*α* level compared to the control value was noticed only after *E*3 (*P* < 0.001); however, the tendency to increase in the level of 8-epi PGF2*α* was noticed with each subsequent exposure. The level of 8-epi PGF2*α* after *E*3 was also significantly higher compared to its value after *E*1 (*P* < 0.05). After second and third exposures to EMF of 7 mT, the significant increase of 8-epi PGF2*α* level relative to 1 mT was noticed (*P* < 0.001).

### 3.3. Comparison between Basal Level and Open Field Test-Induced Level of Oxidative Stress Markers

Table 2 presents the results of analysis comparing the basal levels of oxidative stress markers to their levels after the open field test for each group, respectively: C/B vs .C/OF, EMF/B/1mT vs. EMF/OF/1mT, and EMF/B/7mT vs. EMF/OF/7mT). The analysis showed that both the open field test and the number of exposures do not affect the CP level in the control group, only interaction of both factors had a significant influence on CP level in this group (Table 2(a)). In the group exposed to EMF of 1 mT, the CP level has been changed after open field, and the interaction between the open field test and the number of exposures also profoundly affected the CP level (Table 2(b)). In the group exposed to EMF of 7 mT, we have found the significant influence of the open field test on the increase in CP levels, and the number of exposures has no effect; however, the interaction between these factors was significant (Table 2(c)). The changes of 8-epi PGF2*α* level in the control group were dependent only on the number of exposures (Table 2(d)). The clearest effect of both factors as well as the interaction between them was noticed in rats exposed to EMF of 1 mT (Table 2(e)). In rats exposed to EMF of 7 mT, the 8-epi PGF2*α* level was not affected by any factor (Table 2(f)).

Valuable results were received when we evaluated the percentage changes in the level of stress markers in comparison to their level in the control C/B group separately after each exposure (set at 100%: reference value) (Figure 5).

CP level in the prefrontal cortex (Figure 5(a)) in group C/OF increased clearly after *E*3 (by 64%) in comparison to the C/B group. In the EMF/B/1 mT group, the level of CP was higher by 117% than that in the control group (C/B) after *E*3. Otherwise, after exposure to open field, the level of CP in rats previously exposed to EMF of 1 mT in comparison to the level in the EMF/B/1mT group was increased only after *E*1 (by 45%) and then was decreased even in comparison to both control groups (C/B and C/OF). In EMF/B/7mT, the level of CP after each subsequent exposure was higher in comparison to the value in the control group (C/B) (by 50 51 and 79%, respectively) and the open field test remarkably increased the level of the parameter after *E*1 (by 118%) and *E*3 (by 168%), except after *E*2 when the value of CP was similar to its basal level.

A similar direction of changes as in the case of CP groups level was observed in 8-epi PGF2*α* level in the control group as well as in groups exposed to EMF of 1 and 7 mT (Figure 5(b)). In the case of 8-epi PGF2*α* in animals exposed to EMF of 7 mT, the higher basal level of this marker should be noticed after each exposure in comparison to the control level (C/B) with its incredibly high level after *E*3 (267% of reference value). After OF test, the level of 8-epi PGF2*α* decreased slightly relative to its basal level in this group.

### 3.4. The Basal Level of Total Antioxidant Capacity (TAC)

The intensity of EMF, as well as EMF intensity × number of exposures interaction, had a significant influence on TAC level (Table 3(a), Figure 6(a)). The level of TAC in animals exposed to EMF of both intensities was not significantly different from that noticed in the C/B group. In the group exposed to EMF of 1 mT, only after *E*3 the tendency to decrease in the TAC level in comparison to the control value was observed. The only detectable decrease of TAC level in the EMF/B/1mT group was observed after *E*3 relative to that after *E*2 (*P* < 0.05). The TAC level in animals exposed to EMF of 7 mT was lower than that in the EMF/B/1mT group after *E*2 (*P* < 0.05). However, the tendency to decrease in the value of TAC level in animals exposed to EMF of 7 mT was observed after each subsequent exposure relative to its level in the C/B group.

### 3.5. The Open Field-Induced Level of Total Antioxidant Capacity (TAC)

The direction of changes in the open field test-induced level of TAC in all groups was similar as in the case of its basal level. The strength of the electromagnetic field, as well as the number of exposures, significantly influenced the changes of open field-induced TAC level. The interaction between both factors was also notable (Table 3(b), Figure 6(b)). After a single exposure to EMF of 1 mT, the TAC level was higher compared to the value in the respective control group (C/OF) (*P* < 0.05). After *E*2, the value of TAC was comparable to the control level, and only after *E*3, it dropped significantly compared to the value in the control group (*P* < 0.05). In addition, in the EMF/OF/1mT group, the TAC level after *E*1 and *E*2 was clearly higher compared to that observed after *E*3 (*P* < 0.001). After first exposure to EMF of 7 mT, the level of TAC was significantly decreased compared to that in control animals exposed to OF (C/OF) (*P* < 0.01) as well as to its value in the EMF/OF/1mT group (*P* < 0.001). Moreover, in the EMF/OF/7mT group, the level of TAC was significantly decreased after *E*1 and *E*3 compared to that noticed after *E*2 (*P* < 0.01).

### 3.6. Comparison between Basal Level and Open Field Test-Induced Level of TAC

Any of the factors did not affect the TAC level in the control group (Table 4(a)). In the group exposed to EMF of 1 mT, the significant influence of the open field test and the number of exposures as well as their interaction on TAC level was found (Table 4(b)). In the 7 mT group, the number of exposures had a significant impact on TAC level. Moreover, the interaction between the open field test and the number of exposures was also significant (Table 4(c)).

The percentage changes in TAC level (Figure 7) in the control group after the open field test was clear. The value of antioxidant's level marker was increased in comparison to its basal level after *E*1 by 17%. In the EMF/OF/1mT group, the TAC amount was higher than that in the EMF/B/1mT group after *E*1 (by 45%) and *E*2 (by 15%), while after *E*3, the TAC level was close to its basal level. In rats from the EMF/B/7mT group after all exposures, the basal level of TAC was lower than that in the C/B group (by 13, 20, 3%, respectively). In the EMF/OF/7mT group, the noticed value of TAC after *E*1 was similar to the basal control value; after *E*2, the level of TAC was increased (by 24%); and then, after *E*3, the OF-induced level of TAC was decreased by 15% in comparison to values in EMF/B/7mT.

## 4. Discussion

Our experiments have shown that repeated exposure to the extremely low-frequency electromagnetic field (EMF) profoundly changes the oxidative/antioxidative status in the prefrontal cortex of rats in the EMF intensity- and number of exposure-dependent manner. The level of oxidative stress markers and antioxidants in rats exposed to EMF of 1 mT was not very different from the control value. In rats exposed to EMF of 1 mT, a significantly increased protein carbonyl groups level was noticed only after third exposure compared to the control group. In the case of 8-isoprostanes, the exposure to EMF of 1 mT did not significantly affect their level; however, the tendency to decrease with each following exposure was noticed. Moreover, in the 1 mT EMF-exposed group, the profound change in the basal TAC level was not found. The level of TAC was a little, not significantly increased after the first and second exposures.

Generally, most research confirmed the antioxidative effects of EMF of ≤ 1 mT. Patruno et al. [12] observed elevated catalase (CAT) activity in cell culture (myelogenous leukemia cells: K562) after exposure to 50 Hz 1 mT EMF concomitantly with a decrease in the activity of inducible nitric oxide synthase (iNOS). In an animal model of Huntington's disease EMF (60 Hz and 0.7 mT), exposure reduced levels of oxidative stress biomarkers [27]. In C2C12 muscle cells, no change in reactive oxygen species (ROS) production was observed after exposure to EMF of 1 mT [11]. The research indicating that even low levels (≤ 1 mT) of a single EMF exposure can cause an increase in oxidative stress [10, 28] can also be found. However, in the mentioned in vitro studies, the cells were treated with EMF continuously from 30 min to 24 h, or in animals, the procedure included the one, 21-day lasting period with EMF exposure 4 h/day. It is also important that the duration of exposure also determines the effect of EMF. In Caco 2 cells treated with 50 Hz EMF of 1 mT for 24 h, 48 h, or 72 h, the longer the exposure time, the greater level of oxidative stress was found [29]. It has been also shown that the long-term exposure to the extremely low-frequency magnetic field (100 and 500 *μ*T) 2 h/day for 10 months caused a decrease in the activity of the antioxidant enzyme catalase (CAT). However, the TAC level was lower in the group exposed to 500 *μ*T, and at the same time, in this group, the levels of oxidative stress markers, MDA and MPO (myeloperoxidase), as well as values of total oxidant status (TOS) and oxidative stress index (OSI), were significantly higher [30]. Concerning the risk of development of neurodegenerative disorders after EMF exposure, it is also important that neither 100 nor 500 *μ*T extremely low-frequency magnetic field altered beta-amyloid protein level significantly [31]. It confirms the dose-dependent action of EMF.

Our results showed that EMF of 1 mT creates weak changes in oxidative status in the rat's brain. Many studies showed that stress induces the disruption in homeostasis [15, 32], and as a consequence, an overcompensation response is triggered to reestablish homeostasis, and such effect was seen in response to EMF of 1 mT after two first exposures. The compensatory mechanisms driven during first exposure to EMF seem to be able to maintain the oxidative equilibrium even after the second exposure, only after the third exposure the cumulative effect of all exposures as an increase in oxidative stress simultaneously with a discrete decrease of antioxidants was visible.

In animals exposed to EMF of 7 mT, the characteristic of changes in oxidative stress and antioxidative defence markers was quite different. The clear increase of CP groups was visible earlier than in the group exposed to EMF of 1 mT— already after the second exposure and remained high after the third exposure. Moreover, the tendency to increase in the level of 8-epi PGF2*α* with each subsequent exposure was noticed, and eventually, after *E*3, the 8-epi PGF2*α* level was significantly higher (more than 2.5 times) than that in the control group. In animals exposed to EMF of 7 mT, the tendency to decrease in the TAC level was observed after each subsequent exposure relative to its level in the control group. The present results indicate that the changes in TAC level were accompanied by a parallel increase in oxidative stress markers. The other research also showed that exposure to EMF (40-50 Hz) of intensities close to this used in our research (≥ 6 mT) alters oxidative stress and antioxidant defense parameters. In the serum of ICR mice, the level of MDA was significantly higher after exposure to EMF of 6, 8, and 10 mT, and simultaneously, the level of antioxidant enzyme superoxide dismutase (SOD) activity was decreased [8]. Similarly, in mouse brains subjected to EMF (8 mT), the levels of MDA, ROS, nitrogen oxide (NO), and nitric oxide synthase (NOS) were increased, whereas activities of antioxidants enzymes: SOD, CAT, and glutathione peroxidase (GPx), were decreased [33]. The disturbance of oxidative status was also found in testes of rats (diabetic model) exposed to EMF (8.2 mT) in the form of elevated MDA and NO levels and diminished glutathione (GSH) level was found [34]. The measurements of oxidative stress markers in the rat's heart and plasma after exposure to EMF of 7 mT showed a significant increase in thiobarbituric acid reactive substances (TBARS) and H_2_O_2_ concentration and the diminished antioxidant defense decreased TAC, GSH, and total free thiol groups level [20]. In vitro studies confirmed that after exposure to electromagnetic field (8 mT), a decrease in the viability and morphological changes of the rat hippocampal neurons were observed with an increase in the level of MDA and ROS and a decrease in the activity of SOD [22]. Otherwise, opposite results have also been received, e.g., poststroke patients after EMF therapy (7 mT) showed improved enzymatic antioxidant activity [13]. As in the case of studies on the effects of EMF of lower intensities ≤ 1 mT, the abovementioned results are the consequence of continuous exposure for 14-28 days (day by day, 15 min-4 h/day) or as in the case of in vitro studies— one 90-min lasting treatment. The present results indicate that in such challenging stress situations as repeated exposure to EMF of 7 mT, the balance is disturbed in the direction of a higher level of oxidative stress. It also suggests that not all homotypic stressors cause response habituation. Responses to more "severe" stressors are maintained over time, perhaps due to the higher costs required to adapt to the particular situational demand [16]. Thus, the cumulative effect of repeated exposure to EMF of high intensity resulted in increased oxidative stress.

In our research, we identified the directions and dynamics of some mechanisms that may be brought into play in EMF-provoked changes. Although moderate stimulation by EMF (1 mT) even repeated might be not demanding for the organism, if strong (7 mT), it can lead to deleterious effects due to the increase in oxidative stress. The integrative processes between all “players” determining oxidative/antioxidative balance appear to determine the final effect of EMF [2, 15]. As a result, even subtle changes in the brain can change the function of the neuronal circuits. An undisturbed oxidative/antioxidative balance is essential for the normal function of the organism. Unbalanced concentrations of oxidative processes products decrease the chance of overcompensation and increase brain vulnerability to other potentially dangerous events.

We have found that the exposure of rats to EMF of 1 mT influenced the oxidative/antioxidative status evolved in response to subsequent (heterogenous in relation to EMF) stress factor—open field test. EMF of 1 mT diminished the response to another stressor as the small elevation of open field-induced CP concentration was visible only after the first exposure to EMF, each next period of EMF-treatment decreased the level of the marker. In the case of 8-isoprostanes, their level was diminished after two first exposures, and after E3 received a similar value as in the respective group not-exposed to OF. In 1 mT EMF-treated rats, the augmented antioxidant defense in response to a new stress factor was visible after first exposure; then, the adaptation as the decrease in TAC level was observed. The changes in the TAC level can partly explain the reduction in oxidative stress in this group. Our results allowed us to conclude that the subtle changes in the level of oxidative status in animals repeatedly exposed to EMF of 1 mT were enough to change the profile of oxidative processes after exposure to another kind of stress factor— open field test. It suggests that it can be a kind of habituation, when one stressor diminishes the response to the second one [16].

The EMF of 7 mT disturbs the oxidative/antioxidative balance as the changes in oxidative stress markers as well as antioxidant capacity level were still clear after each subsequent exposure to the open field. The pattern and size of the changes in 8-epi PGF2*α* level after subsequent exposures to open field in rats previously exposed to EMF of 7 mT were close to the changes in basal level. The open field-induced CP level in rats exposed to EMF of 7 mT has been increasing with each subsequent exposure and was definitely higher than that in respective control as well as in the 1 mT EMF-exposed group. The response to first contact with a new stressor was also the significant decrease in TAC level, which then increased to the value not different from that in the respective control group. Thus, we suggest that the exposure to one stressor (EMF) sensitizes the organism to a second stressor (open field), resulting in a faster onset of oxidative stress and its higher level in 7 mT exposed animals in comparison to the values in 1 mT EMF-treated rats. Djordjevic et al. [35] have also found that in rats exposed to open field after EMF exposure (50 Hz, 10 mT, 24 h for 7 days) the levels of superoxide anion and nitrites in the hypothalamus were increased compared to the control group; however, the observed changes are the synergic effect of both factors, as the oxidative status of rats after EMF exposure was not evaluated in this research. Our results suggest that a high level of magnetic flux density (7 mT) of EMF is able to disturb the brain oxidative/antioxidative status, and to shift its set-point in the direction of increase of oxidative processes and as a consequence can augment the oxidative processes in response to the next stress events.

## 5. Conclusions

Summarizing, as we hypothesized, the level of EMF appears to be essential for direction and dynamics of the stress response: changes in oxidative/antioxidative parameters after exposure to 1 mT EMF were observed at a lower level than these after exposure to 7 mT EMF; moreover, the character of changes was also different. Our data confirmed that the exposure to EMF of 1 mT can establish a new “set-point” for cellular oxidative processes and may initiate cellular adaptation by activation of intrinsic signaling pathways directed into the decrease of oxidative stress, although the cumulative effect of repeated exposure cannot be definitely excluded. Otherwise, in the case of a stronger electromagnetic field (7 mT), the adaptive processes are not sufficient to counteract its detrimental effects. Consequently, EMF can change the vulnerability of the organism to subsequent stress factors and thus to diseases, mainly related to the nervous system. Our research for the first time showed the different “mode of action” of EMF in relation to oxidative/antioxidative status in the brain dependently on its magnetic flux density value. In addition, what is even more important, we proved that the effects of EMF can be permanent and influence the response of the organism to other stress events and in this way modulate the vulnerability to the diseases. We are convinced that the results of our research extended the knowledge on mechanisms of EMF's impact on human health. Further, the elucidation of the EMF-induced changes in the oxidative/antioxidative status is necessary to a reliable assessment of the influence of EMF on the brain. The obtained results can also provide a new view on possible therapeutic properties of the magnetic field as well as a new direction in the risk assessment of EMF exposure. As the 1 mT seems to have a potentially protective impact on the brain, the studies are worth continuing.

## Figures and Tables

**Figure 1:** The plot of the mean value of magnetic flux density within the area of the animal's cage in the coil. Abbreviations: *B*: magnetic flux density vector, *B*/*B*0: normalized magnetic flux density relative to the value in the geometrical centre of the coil; *z*/*l*: normalized distance from the coil centre along *z*-axis; *x*/2*r*: normalized distance from the solenoid centre along *x*-axis; *l*: coil length; *r*: coil radius

**Figure 2:** Experimental design. (a) First set of experiments: assessment of basal level of oxidative stress markers and antioxidants. (b) Second set of experiments: assessment of open field-induced level of oxidative stress markers and antioxidants.

**Figure 3:** The basal level of oxidative stress markers: (a) CP groups and (b) 8-epi PGF2*α* in the prefrontal cortex of rat's brain. Animals were exposed once to three times (*E*1-*E*3) to EMF of 1 or 7 mT or control conditions. Values are presented as mean ± SEM. The lines show the direction of changes in the level of stress markers in 1 mT (dotted line) and 7 mT (solid line) groups after each subsequent exposure. Statistically significant differences between animals from the same group are denoted ^##^*P* < 0.01 and ^###^*P* < 0.001; and these between experimental groups are denoted ^∗∗∗^*P* < 0.001.

**Figure 4:** The open field-induced level of oxidative stress markers: (a) CP groups and (b) 8-epi PGF2*α* in the prefrontal cortex of rat's brain. Animals were exposed once to three times (*E*1-*E*3) to EMF of 1 or 7 mT or control conditions. Values are presented as mean ± SEM. The lines show the direction of changes in the level of stress markers in 1 mT (dotted line) and 7 mT (solid line) groups after each subsequent exposure. Statistically significant differences between animals from the same group are denoted ^#^*P* < 0.05 and ^###^*P* < 0.001, and these between experimental groups are denoted ^∗^*P* < 0.05 and ^∗∗∗^*P* < 0.001.

**Figure 5:** Percentage changes in the basal level as well as open field-induced level of oxidative stress markers: (a) CP groups and (b) 8-epi PGF2*α* in each experimental group in relation to their level in the control C/B group set at 100% after each subsequent exposure (*E*1-*E*3).

**Figure 6:** The basal (a) and open field-induced level of TAC (b) in the prefrontal cortex of the rat's brain. Animals were exposed once to three times (*E*1-*E*3) to EMF of 1 or 7 mT or control conditions. Values are presented as mean ± SEM. The lines show the direction of changes in the level of TAC in 1 mT (dotted line) and 7 mT (solid line) groups after each subsequent exposure. Statistically significant differences between animals from the same group are denoted ^#^*P* < 0.05, ^##^*P* < 0.01, and ^###^*P* < 0.001, and these between experimental groups are denoted ^∗^*P* < 0.05, ^∗∗^*P* < 0.01, and ^∗∗∗^*P* < 0.001.

**Figure 7:** Percentage changes in the basal level as well as open field-induced level of TAC in each experimental group in relation to their level in control C/B group set at 100% after each subsequent exposure (*E*1-*E*3).

**Table 1:** Results of statistical analysis of the oxidative markers concentrations in the prefrontal cortex.

	Dependent variable	Effect	*df*	*F*	*P*
a	CP basal level	Intensity of the electromagnetic field (mT)	2	22.133	*<0.001*
		Number of exposures (*E*1‐*E*3)	2	16.681	*<0.001*
		(mT) × (*E*1‐*E*3)	4	9.851	*<0.001*
		Error	68		
b	8-epi PGF2*α* basal level	Intensity of the electromagnetic field (mT)	2	15.231	*<0.001*
		Number of exposures (*E*1‐*E*3)	2	0.191	0.827
		(mT) × (*E*1‐*E*3)	4	2.343	0.063
		Error	73		
c	Open field-induced CP level	Intensity of the electromagnetic field (mT)	2	190.737	*<0.001*
		Number of exposures (*E*1‐*E*3)	2	19.793	*<0.001*
		(mT) × (*E*1‐*E*3)	4	12.051	*<0.001*
		Error	71		
d	Open field-induced 8-epi PGF2*α* level	Intensity of the electromagnetic field (mT)	2	13.921	*<0.001*
		Number of exposures (*E*1‐*E*3)	2	0.657	0.522
		(mT) × (*E*1‐*E*3)	4	7.753	*<0.001*
		Error	66		

F: GLM; statistically significant *P* value: indicated in italic; CP: protein carbonyl groups.

**Table 2:** Results of statistical analysis of effects of open field stress on oxidative stress markers level in relation to its basal level in each experimental group.

	Dependent variable/group	Effect	*df*	*F*	*P*
a	CP Control group	Open field effect	1	1.964	0.168
		Number of exposures (*E*1-*E*3)	2	2.253	0.118
		Number of exposures × open field effect	2	32.078	*<0.001*
		Error	42		
b	CP EMF/1mT	Open field effect	1	52.023	*<0.001*
		Number of exposures (*E*1-*E*3)	2	3.077	0.055
		Number of exposures × open field effect	2	66.370	*<0.001*
		Error	49		
c	CP EMF/7mT	Open field effect	1	47.966	*<0.001*
		Number of exposures (*E*1-*E*3)	2	1.876	0.164
		Number of exposures × open field effect	2	12.193	*<0.001*
		Error	48		
d	8-epi PGF2*α* Control group	Open field effect	1	2.995	0.091
		Number of exposures (*E*1-*E*3)	2	33.444	*<0.001*
		Number of exposures × open field effect	2	1.422	0.252
		Error	44		
e	8-epi PGF2*α* EMF/1mT	Open field effect	1	14.228	*<0.001*
		Number of exposures (*E*1-*E*3)	2	15.181	*<0.001*
		Number of exposures × open field effect	2	6.000	*0.005*
		Error	47		
f	8-epi PGF2*α* EMF/7mT	Open field effect	1	2.005	0.163
		Number of exposures (*E*1-*E*3)	2	2.649	0.081
		Number of exposures × open field effect	2	0.064	0.938
		Error	48		

F: GLM; statistically significant*P*value: indicated in italic; CP: protein carbonyl groups.

**Table 3:** Results of statistical analysis of the TAC level in the prefrontal cortex.

	Dependent variable	Effect	*df*	*F*	*P*
a	TAC basal level	Intensity of the electromagnetic field (mT)	2	5.088	*0.008*
		Number of exposures (*E*1-*E*3)	2	2.209	0.117
		(mT) × (*E*1-*E*3)	4	3.163	*0.018*
		Error	79		
b	Open field-induced TAC level	Intensity of the electromagnetic field (mT)	2	11.803	*<0.001*
		Number of exposures (E1-E3)	2	27.075	*<0.001*
		(mT) x (E1-E3)	4	11.086	*<0.001*
		Error	78		

F: GLM; statistically significant*P*value: indicated in italic; TAC: total antioxidant capacity.

**Table 4:** Results of statistical analysis of effects of open field stress on TAC level in relation to its basal level in each experimental group.

	Dependent variable/group	Effect	*df*	*F*	*P*
a	TAC Control group	Open field effect	1	1.375	0.246
		Number of exposures (*E*1-*E*3)	2	0.568	0.570
		Number of exposures × open field effect	2	0.905	0.411
		Error	52		
b	TAC EMF/1mT	Open field effect	1	12.290	*<0.001*
		Number of exposures (*E*1-*E*3)	2	39.426	*<0.001*
		Number of exposures × open field effect	2	12.297	*<0.001*
		Error	52		
c	TAC EMF/7mT	Open field effect	1	2.301	0.135
		Number of exposures (*E*1-*E*3)	2	7.958	*<0.001*
		Number of exposures × open field effect	2	13.983	*<0.001*
		Error	53		

F: GLM; statistically significant*P*value: indicated in italic; TAC: total antioxidant capacity.

## Data Availability

The data used to support the findings of this study are included within the article.
